# To Investigate the Effect of Magnetic Resonance Imaging (MRI) and Diffusion Tensor Imaging (DTI) in the Diagnosis of Mild Craniocerebral Injury

**DOI:** 10.1155/2022/8469939

**Published:** 2022-09-21

**Authors:** Xiaoyan Lei, Dan Qin, Gangming Zhu

**Affiliations:** ^1^Department of Radiology, Hainan General Hospital, Affiliated Hainan Hospital to Hainan Medical University, Haikou, Hainan, China; ^2^Department of Radiology, Beijing Rehabilitation Hospital, Capital Medical University, Beijing, China; ^3^Department of Radiology, Dongguan Songshan Lake Tungwah Hospital, Dongguan, Guangdong, China

## Abstract

In order to assess the value of magnetic resonance imaging (MRI) and diffusion tensor imaging (DTI) in microscopic brain scans. Diffusion tensor imaging (DTI) and magnetic resonance spectroscopy (MRI) changes over time in patients with traumatic brain injury (TBI) show a relationship between recovery from coma and overall Glasgow prognostic parameters. The value of DTI combined with MRI in evaluating TBI has been investigated. 10 patients with TBI received 10 evaluations of magnetic resonance imaging, DTI and MRI scans. Thalamic plate nucleus, reticular nucleus, and retinal developmental activity were measured in normal controls and TBI coma (2-3 weeks) and mild (>4 weeks) patients. Anisotropy, mean diffusion coefficient, axial diffusion coefficient, and radial diffusion coefficient were measured using MRI together with acetylaspartic acid, choline, creatinine, and lactic acid. Independent control *t*-tests were conducted between controls and TBI patients, and 1-test paired between moderate and severe injuries, and regression and correlation were evaluated. Evaluated for all measures and treatments. DTI and MRI scores in TBI patients differed from normal controls. DTI and MRI can predict the prognosis of TBI patients better. The limitations of the thalamus-retinal activation system are gradually restored. axial diffusion coefficient and radial diffusion coefficient can be used to evaluate the reliability of comatose patients with TBI. DTI and MRI scans of the patient's brain can predict recovery and guide treatment in TBI coma patients.

## 1. Introduction

Cranial brain injury is a common neurosurgery traumatic disease, of which 70%~90% are mild to the brain injury, most of which are reversible forgetting, transient loss of consciousness, and other symptoms, which seriously affect the life, study, and work of patients [1]. However, due to the low positive rate of mild craniocerebral injury in skull, CT and conventional magnetic resonance imaging (MRI) examination and the lack of attention to neurosurgery, it is easy to cause the development of the disease and even lifelong disability. Therefore, early diagnosis and treatment of mild brain injury is particularly important to improve patient prognosis. With the continuous improvement of imaging technology, clinicians have deepened their understanding of mild craniocerebral injury, and magnetic resonance diffusion tensor imaging is used in diagnosis mainly by analyzing the amount of water molecules in the brain [2]. MR diffusion tensor imaging (diffusion tensor imaging, DTI) is a new MRI scanning technology that has been used clinically for many years that describes the distribution of water molecules in the clinic, which can measure and measure the movement of water molecules in the brain tissue.  Figure 1 shows the composition of magnetic resonance imaging system. Cranial brain injury is a common neurological disease in clinical medicine, which is a common traumatic condition caused by external factors. It mainly refers to that, under the action of external forces, injury to the human scalp, skull, and brain tissue. The clinical manifestations are cognitive difficulties, the difficulty of somatic action, the disease easily leads to mental abnormalities, brain edema, and other symptoms. When scanning for the clinically commonly used CT and MRI, the scan positive rate was low, because the inspection was not comprehensive enough. In the clinicians, often paying insufficient attention to the condition, misdiagnosis and missed diagnosis often occur, if the patient does not receive timely and effective treatment, it can easily be life-threatening [3]. With the continuous development of medical science and technology, application in the diagnosis of brain injury is more and more accurate, including magnetic resonance as one of the main means of clinical detection. It can help doctors for the movement of brain tissue molecules, help improve the accuracy of brain patients, and applied in the diagnosis of brain injury is very common.

## 2. Literature Review

In view of this research problem, Xiao et al. performed DTI scans in some patients with mild brain injury and detected elevated ADC values in some areas, which is different from the results of this study, and may be related to the study subjects in different periods after trauma at the time of testing. In the DTI scan, the FA value detection can reflect the brain tissue damage in patients with mild brain injury more strongly than the ADC value [4]. Ni et al. found that no abnormal signals were found in routine MRI and DTI scans of patients with mild brain injury, and the ADC values of bilateral frontal white matter, internal capsule and corpus callosum were not compared with healthy people (controls), and the FA value was significantly lower than that of the control group (*P* < 0.05) [5]. Significant diffuse hypersignaling in the cerebral gyrus cortex with reduced ADC values in the occipital lobe was observed by Zhang et al.. Follow-up observed brain atrophy in this area and low signal on DTI. they suggest that DTI can be used to locate epileptic foci and predict prognosis. The DTI has the potential to reflect part of the pathological changes in epilepsy, and its results can guide the accurate conduct of surgical procedures, and thus affect the prognosis of epilepsy patients [6]. Azorin et al. evaluated the application value of DTI in the diagnosis of CNS diseases, compared the FA and ADC values of different diseases, and summarized the diagnostic experience [7]. Pak et al. found that whole-brain CHO/Cr was associated with prognosis, and this study also found a negative relationship between CHO/Cr in chronic-stage ARAS in patients and prognosis [8]. Gattringer et al. analyzed the effect of magnetic resonance diffusion imaging in central system diseases [9]. Li et al. found that in acute cerebral infarction, a large number of water molecules enter the cells, resulting in intracellular edema and reduced diffusion of water molecules inside and outside the cells, resulting in reduced free diffusion of total water molecules at the ischemic site, swelling of white matter fiber bundles at the infarct site, limited movement of water molecules, increased diffusion anisotropy, and increased FA value [10]. Hong et al. found that the angiogenesis of malignant brain tumors is more than that of benign tumors, and the density of tumor cells in the parenchyma is also relatively large. In addition, due to the limitation of biofilm structure and the adsorption of macromolecular substances on water molecules, there is an obstacle to the diffusion of water molecules. ADC increased significantly and FA value decreased, indicating that DTI is closely related to the severity of leukoaraiosis [11]. Thia et al. found that in multiple sclerosis, DTI can quantitatively and noninvasively evaluate the demyelinating plaque in the brain and the damage degree of normal white matter on conventional MRI. The changes of Fa value of MS lesions in different periods have their own characteristics. The accumulation of inflammatory cells and myelin disintegration products potentially limits the diffusion of water molecules, forming a diffusion barrier without directional water molecules, resulting in the decrease of FA value [12]. Giordano et al. found that DTI imaging technology has characteristics of brain endoplasmic injury in toxic encephalopathy. Compared with the control group, FA in the corpus callosum and corpus callosum decreased significantly [13].

According to the current study, the combined examination can better the role of MRI in mental illness. In this study, MRI changes in comatose patients showed decreased NAA/Cr and NAA/CHO but increased CHO/Cr in the acute phase. NAACR in the ARAS and NAA/CHO and CHO/Cr in the thalamus were not different from normal controls in the small period. This confirmed the results of the DTI analysis done in this study, i.e., the slow recovery of the ARAS unlike the thalamus can explain the long-term memory loss after the brain injury. This study found a negative relationship between CHO/Cr and clinical outcomes in ARAS patients.

## 3. Method

### 3.1. Case Selection

10 TBI patients (5 men and 5 women) with different levels of consciousness and hospitalized for more than two weeks were selected, with an average age of 45.5 years (Table 1). In the human population, patients should stabilize all vital signs and treatment in neurosurgery within 72 hours of craniocerebral injury to eliminate bias due to treatment is different. In the normal control group, healthy subjects (5 males and 5 females) were matched for patient age, sex, and education level, with mean age between 48.0.

Patients with the following conditions will be excluded: (1) patients with previous history of nervous system diseases; (2) patients with trauma complicated with hypoxemia; and (3) patients with contraindications to magnetic resonance examination, such as metal foreign bodies or implants in the body.

### 3.2. Data Acquisition

The enrolled patients underwent imaging examination in the acute stage (the second week after admission) and mild stage (the fourth week after admission and later), and the recovery of the patients was evaluated in the recovery stage (three months after discharge). Healthy people in the normal control group were selected for only one imaging examination. Imaging examination included routine MRI and DTI. Data collection were as follows: whole brain examination was performed with GESignaExciteHD1.5 T superconducting magnetic resonance scanner. The scanning sequence included T_1_WI (TR/TE = 400 ms/15 ms); T_2_WI (TR/TE = 3000 ms/100 ms); DTI (TR/TE = 10000 ms/95 ms, Matrix = 128∗128, FOV = 24, layer thickness = 4 mm, and layer spacing = 0 mm); and MRI (TR/TE = 10000 ms/95ms, Matrix = 128^∗^128, FOV = 24, layer thickness = 4 mm, and layer spacing = 0 mm. Magnetic field intensity = 500 T/m, Gradient switching rate = 150 mT/ms, TR/TE = 5000 ms/980 ms, layer thickness = 5 mm, and layer spacing = 1.0 mm). Locate and draw four brain regions on T1 through FSLv.5.0: thalamic lamina nucleus, reticular nucleus, and ARAS related brain regions (pons medulla oblongata). Each region of the brain draws its region of interest three times and sends the generated region of interest into the ADW4.4 workspace. Functool software combined with DTI line data after processing to measure and obtain FA, MD, Da, and Dr of the region of interest and obtain the average of the three values of the region of interest. The changes in NAA, Cr, CHO, and Lac in four regions of the brain were measured by MRI. Image data integration and quality control were performed by two radiologists [14].

### 3.3. Follow-Up Data Collection

Follow up of the enrolled patients was arranged, and both CRS-R and GOS-R were used to assess the prognosis during the review of the hospital outpatient clinic 3 months after the injury.

### 3.4. Statistical Analysis

The data in the study were analyzed and processed using SPSS 20.0 software, and the count data were represented by the rate (%) and the measurement data by (*t*). If *P* < 0.05, the test was statistically significant [15].

## 4. Results and Analysis

### 4.1. DTI Analysis

1. In the comparison between acute phase and light phase, FA in light phase was higher than that in acute phase, and MD in light phase increased [16]. Compared with the acute phase, DA in reticular nucleus and plate nucleus recovered in light. No significant difference was found between pons and medulla oblongata. DR in the four regions of interest decreased significantly.  Table 2 shows the results of paired *t*-test of acute phase and light DTI parameters in each region of interest
2. Compared with the normal control group, FA and MD were lower in the acute and mild stages than in the normal control group, but there was no difference between FA and normal control in the thalamus small amount of interest, and MD remains the same. Lower than that of the normal control group. Da decreased significantly in the acute phase. In the small form, the pons and core elongation were lower than in the normal control group. During acute illness, Dr was significantly increased in four regions of interest, while thalamic Dr was not significantly different between dementia patients and normal controls.  Table 3 and Figure 2 show the independent sample *t*-test results for DTI lesions of severe and mild disease for each region of interest and the normal control group [17].
3. Correlation analysis between DTI parameters and clinical data through correlation analysis with clinical scores in convalescent stage, it was found that there was no correlation between FA in pons and medulla oblongata in acute stage, MD in thalamus, and CRS-R and mGOS in convalescent stage. But in mild stage, their correlation with clinical consciousness score was obvious (Tables 4–7). In addition, other parameters (Da and Dr) showed good correlation with CRS-R and mGOS in acute stage and mild stage

### 4.2. MRI Analysis

1. In the acute phase, there is a significant difference between NAA/CHO (except NAA/CHO in pons) and light, and there is no difference between NAA/Cr and light in pons and medulla oblongata in the acute phase (Table 8). In this study, only 1 case had Lac peak, which was in plant survival state at the time of follow-up, because there was only 1 case, and this parameter was not included in the subsequent analysis. In MRI methods, all patients underwent a brain MRI examination using a Siemens 1.5 T superconducting MRI scanner (an 8-channel head coil) within 1 week after the injury. Routine T_1_WI, T_2_WI, T_2_-FLAIR, and DWI scans performed first. A DTI scan was then performed. Using a single excitation spin echo plane imaging sequence, scan parameters were as follows: *b* value = 1 000 s/mm, TR/TE = 80000 ms/80.8 ms, FOV = 192 mm × 192 mm. Direction number is 15, and the layer thickness is 1.8 mm. No-interval scan, slice 67, the scan ranged from the skull base to the cranial term. The DTI raw images were transferred to the ADW4.3 workstation for postprocessing by Functool 5.4.07 image processing software to construct FA and ADC maps. Regions of interest (ROI) of 15 to 20 m m in the frontal white matter, temporal white matter, medial capsule, and corpus callosum were selected to measure the FA and ADC values of the selected areas. The measured values were also used for between-group and within-group comparisons
2. Compared with the normal control group, NAA/Cr and NAA/CHO were decreased in the acute phase, while CHO/Cr was significantly increased (Table 9 and Figure 3 [18]. In the acute phase, MRI did not differ from the normal control group. However, there was no significant difference between NAA/Cr in pons and long brain and NAA/CHO and CHO/Cr in thalamus and normal control group
3. Correlation analysis between MRI parameters and clinical data after the correlation analysis with poor clinical outcomes at follow-up, it was found that CHO/Cr only showed correlation with prognosis in mild brainstem ARAS, and the other two items were correlated with prognosis score in acute stage and mild stage. Except that NAA/CHO in the thalamus in the acute stage did not show significant prognostic correlation, the parameters of other regions of interest showed good correlation with prognosis (Tables 10–12) [19].

### 4.3. Discussion

This study analyzed DTI and MRI parameters in acute and chronic phase with clinical scores of 3 months after injury and found that (1) DTI and MRI parameters can predict recovery and guide treatment in coma TBI patients compared with normal controls [20] (2) DTI and MRI can indicate the prognosis of coma patients with TBI [21] (3) parameter recovery in ARAS is slower than that in the thalamus, and (4) ARAS parameters can better predict the prognosis of coma patients [22]. DTI analysis of patients with TBI coma showed that in the acute phase, the parameters in ARAS and thalamus were significantly different from those of normal controls, but the recovery of the parameters within ARAS was slower than that within the thalamus, and the parameters gradually improved with the stability of the condition during the chronic period. Parameters in the thalamus except MD are basically the same as normal controls, but Da of bridge and medulla is still different from normal controls. Da is in the chronic period, but not in the acute phase, which verifies the important role of ARAS in the maintenance of consciousness. The multiple parts of Da in the system as a parameter of consciousness judgment has very important clinical significance.

Mild brain injury is one of the common traumatic diseases that endanger human health and quality of life [23]. The traditional view is that the patients with mild craniocerebral injury with negative CT and conventional MRI scans have no organic changes in the brain tissue mostly, and the clinical symptoms such as headache and dizziness are mostly caused by neurological disorders. However, some scholars have found that about 15% of patients with mild craniocerebral injury are left with long-term cognitive dysfunction, believing that these patients may have organic lesions of brain tissue. Recent studies have also shown that diffuse axonal injury plays an important role in mild brain injury, especially in the pathological development of the postconcussive syndrome. The cause may be related to the axonal injury caused by the trauma. CT and conventional MRI are common imaging examination methods for craniocerebral lesions, but both examination methods are difficult to reflect the diffusion characteristics and walking direction of brain white matter fibers. DTI is through the detection of water molecule microscopic movement of tissue structure and physiological evaluation of biological changes of MRI check new technology, can not only better reaction to the brain white matter fiber bundle but can also accurately evaluate fiber bundle compression, displacement, infiltration, and other pathological changes, is the spatial directionality of white matter fiber bundle, measure the effective method of water molecule diffusion. FA value is the ratio of the anisotropy component in the diffusion tensor change to the whole expansion amount, and it is also the main indicator of nerve damage such as reaction neuronal deloss, nerve fiber direction change, and myelin demyelination [24]; ADC value is an important indicator of reaction to the type and degree of cerebral edema. Mild craniocerebral injury leads to enlarged periwhite matter space and gliosis, coupled with perivascular damage causing demyelinating changes in nerve tissue. The cellular membrane arrangement of nerve tissue cells in early trauma is disordered and swollen, which increases the diffusion resistance parallel to the axon, which leads to weakened axial diffusion and increased radial diffusion, and reduced diffusion anisotropy features [25, 26].

## 5. Conclusion

This article reviews the effectiveness of magnetic resonance imaging (MRI) diffusion tensor imaging (DTI) in the diagnosis of patients with mild brain tumors. Correlation of DTI and MRI contrast in acute and mild stages with patients' clinical scores 3 months after injury: There was a significant difference in DTI and MRI contrast between the comatose TBI patients and normal controls; Mild DTI and MRI may be prognostic in comatose patients with TBI; Parametric recovery in the ARAS was slower than in the thalamus; and ARAS cannot better predict survival in comatose patients with traumatic brain injury. DTI analysis of TBI comatose patients showed that the abnormalities in the ARAS and thalamus during the acute phase were different from the normal control group, but the abnormalities in the ARAS in the hypothalamus were found to be gradual recovered and those who do not exist at a small level. Except for MD, the difference in the thalamus was essentially the same as that of normal controls, but the difference of Da in the pons and medulla oblongata remained between normal controls. There was a significant difference in Da between mild and normal controls, but no significant difference in the pain level. This confirms the important role of the ARAS in the formation and maintenance of consciousness. In many areas of the body, taking Da as an unconscious decision is an important part of treatment. This study did not analyze all brain data, regardless of the type of injury, and only 10 patients were selected. In future studies, we will add more cases and discuss and analyze the mechanisms of injury so that we can investigate the true nature of comatose TBI patients.

## Figures and Tables

**Figure 1:** Composition of magnetic resonance imaging system.

**Figure 2:** Comparison results of independent sample *t*-test between light DTI parameters of TBI patients and normal control group.

**Figure 3:** Comparison results of independent sample *t*-test between acute phase and light MRI parameters of TBI patients and normal control group.

**Table 1:** Basic information of enrolled patients.

Number	Gender	Age	Damage site	Convalescence	
				CRS-R	mGOS
1	Male	49	Frontal lobe	24	6
2	Male	36	Frontal lobe	24	6
3	Male	67	Frontal lobe, temporal lobe, and parietal lobe	9	3
4	Male	28	Frontal and parietal lobes	14	4
5	Female	55	Occipital lobe and cerebellum	15	4
6	Female	47	Parietal and frontal lobes	11	3
7	Female	48	Thalamus and frontal lobe	10	3
8	Female	34	Parietal and frontal lobes	21	5
9	Male	30	Insula thalamus	8	3
10	Female	51	Frontal and parietal lobes	19	5

**Table 2:** Paired *t*-test of acute and mild DTI parameters.

Region of interest	FA	MD	Da	Dr
Board core	0.04^∗^	0.03^∗^	0.04^∗^	0.04^∗^
Reticular nucleus	0.02^∗^	0.04^∗^	0.04^∗^	0.01^∗^
Pontine	0.03^∗^	0.02^∗^	0.12	0.04^∗^
Medulla oblongata	0.03∗	0.04^∗^	0.23	0.01^∗^

**Table 3:** Independent sample *t*-test of acute and light DTI parameters of TBI patients and normal control group.

Region of interest	Acute phase vs Normal control group				Light vs Normal control group			
	FA	MD	Da	Dr	FA	MD	Da	Dr
Board core	0.04	0.03	<0.01	<0.01	0.09	0.04	0.13	0.30
Reticular nucleus	<0.01	0.03	<0.01	0.03	0.11	0.03	0.21	0.14
Pontine	0.03	<0.01	<0.01	<0.01	0.02	0.02	<0.01	0.01
Medulla oblongata	<0.01	<0.01	<0.01	<0.01	0.03	0.03	<0.01	0.02

**Table 4:** Correlation analysis between FA parameters and CRS-R and mGOS in recovery period.

Parameter	Region of interest	Correlation analysis with CRS-R				Correlation analysis with mGOS			
		Acute stage		Light		Acute stage		Light	
		*R* value	*P* value	*R* value	*P* value	*R* value	*P* value	*R* value	*P* value
FA	Board core	0.16	0.03	0.37	0.02	0.80	0.01	0.36	0.02
	Reticular nucleus	0.20	0.06	0.34	0.02	0.11	0.20	0.22	0.01
	Pons	0.20	0.14	0.46	0.01	0.12	0.29	0.31	0.01
	Medulla oblongata	0.10	0.10	0.27	0.03	0.26	0.09	0.20	0.03

**Table 5:** Correlation analysis between MD parameters and CRS-R and mGOS in recovery period.

Parameter	Region of interest	Correlation analysis with CRS-R				Correlation analysis with mGOS			
		Acute stage		Light		Acute stage		Light	
		*R* value	*P* value	*R* value	*P* value	*R* value	*P* value	*R* value	*P* value
MD	Board core	0.039	0.07	0.48	0.01	0.1	0.09	0.35	0.019
	Reticular nucleus	0.10	0.10	0.30	0.039	0.21	0.16	0.47	0.029
	Pons	0.34	0.019	0.24	0.029	0.66	0.019	0.66	0.01
	Medulla oblongata	0.48	0.019	0.43	0.029	0.77	0.019	0.48	0.01

**Table 6:** Correlation analysis between Da parameters and CRS-R and mGOS in recovery period.

Parameter	Region of interest	Correlation analysis with CRS-R				Correlation analysis with mGOS			
		Acute stage		Light		Acute stage		Light	
		*R* value	*P* value	*R* value	*P* value	*R* value	*P* value	*R* value	*P* value
Da	Board core	0.44	0.04	0.32	0.01	0.44	0.019	0.29	0.03
	Reticular nucleus	0.54	0.01	0.38	0.01	0.53	0.029	0.47	0.03
	Pons	0.41	0.01	0.56	0.02	0.19	0.26	0.45	0.02
	Medulla oblongata	0.26	0.02	0.38	0.02	0.51	0.01	0.38	0.02

**Table 7:** Correlation analysis between Dr parameters and CRS-R and mGOS in recovery period.

Parameter	Region of interest	Correlation analysis with CRS-R				Correlation analysis with mGOS			
		Acute stage		Light		Acute stage		Light	
		*R* value	*P* value	*R* value	*P* value	*R* value	*P* value	*R* value	*P* value
Dr	Board core	0.48	0.01	0.46	0.02	0.42	0.01	0.40	0.03
	Reticular nucleus	0.38	0.02	0.28	0.03	0.33	0.01	0.48	0.02
	Pons	0.46	0.01	0.37	0.01	0.54	0.01	0.20	0.02
	Medulla oblongata	0.40	0.01	0.40	0.01	0.45	0.01	0.45	0.01

**Table 8:** Paired *t*-test of acute and light MRI parameters.

Region of interest	NAACT	NAA/CHO	CHO/Cr
Board core	0.19^∗^	0.02^∗^	0.03^∗^
Reticular nucleus	0.39^∗^	0.01^∗^	0.05^∗^
Pontine	0.05	0.08	0.04^∗^
Medulla oblongata	0.11	0.39^∗^	0.02^∗^

**Table 9:** Independent sample *t*-test of acute phase and light MRI parameters of TBI patients and normal control group.

Region of interest	Acute phase vs Normal control group			Light vs Normal control group		
	NAN/Cr	NAA/CHO	CHO/Cr	NAN/Cr	NAA/CHO	CHO/Cr
Board core	0.04^∗^	0.03^∗^	0.03^∗^	0.02^∗^	0.10	0.07
Reticular nucleus	0.01^∗^	0.03^∗^	0.02^∗^	0.04^∗^	0.08	0.10
Pontine	0.02^∗^	0.02^∗^	0.01^∗^	0.08	0.02^∗^	0.01^∗^
Medulla oblongata	0.02^∗^	0.02^∗^	0.02^∗^	0.09	0.02^∗^	0.03^∗^

**Table 10:** Correlation analysis between NAACR parameters and CRS-R and mGOS in recovery period.

Parameter	Region of interest	Correlation analysis with CRS-R				Correlation analysis with mGOS			
		Acute stage		Light		Acute stage		Light	
		*R* value	*P* value	*R* value	*P* value	*R* value	*P* value	*R* value	*P* value
NAN/Cr	Board core	0.35	0.03	0.14	0.03	0.15	0.03	0.35	0.02
	Reticular nucleus	0.47	0.02	0.20	0.02	0.21	0.01	0.24	0.03
	Pons	0.3	0.02	0.25	0.02	0.14	0.02	0.12	0.03
	Medulla oblongata	0.2	0.02	0.22	0.02	0.16	0.02	0.22	0.01

**Table 11:** Correlation analysis between NAA/CHO parameters and CRS-R and mGOS in recovery period.

Parameter	Region of interest	Correlation analysis with CRS-R				Correlation analysis with mGOS			
		Acute stage		Light		Acute stage		Light	
		*R* value	*P* value	*R* value	*P* value	*R* value	*P* value	*R* value	*P* value
NAA/CHO	Board core	0.05	0.20	0.20	0.01	0.07	0.05	0.22	0.04
	Reticular nucleus	0.07	0.10	0.17	0.01	0.10	0.07	0.23	0.05
	Pons	0.26	0.03	0.24	0.02	0.20	0.03	0.37	0.01
	Medulla oblongata	0.28	0.03	0.21	0.02	0.29	0.03	0.29	0.02

**Table 12:** Correlation analysis between CHO/Cr parameters and CRS-R and mGOS in recovery period.

Parameter	Region of interest	Correlation analysis with CRS-R				Correlation analysis with mGOS			
		Acute stage		Light		Acute stage		Light	
		*R* value	*P* value	*R* value	*P* value	*R* value	*P* value	*R* value	*P* value
CHO/Cr	Board core	0.10	0.09	0.10	0.08	0.12	0.05	0.20	0.08
	Reticular nucleus	0.19	0.06	0.23	0.07	0.08	0.08	0.10	0.13
	Pons	0.38	0.07	0.30	0.29	0.16	0.07	0.43	0.02
	Medulla oblongata	0.07	0.12	0.47	0.19	0.09	0.08	0.38	0.03

## Data Availability

No data were used to support this study.
